# Sustainability of common pool resources

**DOI:** 10.1371/journal.pone.0170981

**Published:** 2017-02-17

**Authors:** Raja Rajendra Timilsina, Koji Kotani, Yoshio Kamijo

**Affiliations:** 1 School of Economics and Management, Kochi University of Technology, Kochi-shi, Kochi, Japan; 2 Research Center for Future Design, Kochi University of Technology, Kochi-shi, Kochi, Japan; 3 College of Business, Rikkyo University, Toshima-ku, Tokyo, Japan; 4 Urban Institute, Kyushu University, Nishi-ku, Fukuoka, Japan; Tianjin University of Technology, CHINA

## Abstract

Sustainability has become a key issue in managing natural resources together with growing concerns for capitalism, environmental and resource problems. We hypothesize that the ongoing modernization of competitive societies, which we refer to as “capitalism,” affects human nature for utilizing common pool resources, thus compromising sustainability. To test this hypothesis, we design and implement a set of dynamic common pool resource games and experiments in the following two types of Nepalese areas: (i) rural (non-capitalistic) and (ii) urban (capitalistic) areas. We find that a proportion of prosocial individuals in urban areas is lower than that in rural areas, and urban residents deplete resources more quickly than rural residents. The composition of proself and prosocial individuals in a group and the degree of capitalism are crucial in that an increase in prosocial members in a group and the rural dummy positively affect resource sustainability by 65% and 63%, respectively. Overall, this paper shows that when societies move toward more capitalistic environments, the sustainability of common pool resources tends to decrease with the changes in individual preferences, social norms, customs and views to others through human interactions. This result implies that individuals may be losing their coordination abilities for social dilemmas of resource sustainability in capitalistic societies.

## Introduction

Capitalism has become a dominant social regime over the last several decades [1]. Economic theory claims that goods and services are “efficiently” produced, allocated and consumed through competitive markets in capitalism, and this efficient property serves as the main engine of economic growth [2]. However, some of these principles do not appear to function in reality as theory predicts. For instance, intra- and inter-generational allocations of environmental goods and natural resources are claimed to be inefficient under capitalistic conditions as illustrated by climate change trends and the depletion of the world’s forests. Thus, resource sustainability has become a key issue of a growing concern in relation to capitalism.

When natural resources are provided as commons, they are typically referred to as common pool resources (hereafter, CPRs). In the CPR allocations, individuals are known to face a coordination problem of social dilemmas and a sustainability problem of depletion [3, 4]. Ostrom [5] states that individuals tend to lose their ability for coordination in social dilemmas unless they are facilitated through communications and monitoring. Interestingly, however, Fruteau et al. [6] have shown that animals such as vervet monkeys overcome social dilemmas without any intervention. It thus remains an open question whether or not humans have coordination abilities to solve the dilemma to sustainably manage CPRs.

Economists have long examined the CPR dilemmas via experimental methods. Walker and Gardner’s paper is a pioneering work in the examination of CPRs in experimental settings [7]. Additional studies have examined CPR games through laboratory experiments that mimic some environments observed in the field (e.g., the probabilistic destruction of the commons and various strategic situations) [8–10]. Decision-making processes and preferences of actual resource users for CPRs have been examined through field experiments [9, 11–13]. All of these field studies have been conducted in static or repeated-game settings, and show that some external devices such as information provisions and other-regarding preferences are essentials to CPR solutions.

Another group of works explicitly incorporates resource dynamics in the CPR experiments and analyzes how the dynamic nature of resources affects the outcomes compared with static or repeated cases [14–17]. These studies have demonstrated that the regeneration processes of CPRs critically affect the sustainability of resource use. From these works, other studies have introduced inter-generational allocation and process uncertainties of resource dynamics, showing that the one-way nature of inter-generations and process uncertainties compromise sustainability [18, 19]. More recent works have theoretically analyzed the dynamics of public resources and people’s cooperation in spatial public goods game [20–24]. These works suggest that reputation, mobility and neighborhood environments are important determinants for solving social dilemmas in a dynamic spatial environment.

Ostrom discusses that individuals can organize sustainable resource use in specific socio-ecological environments that enable interpersonal communication and monitoring [25]. This points to the importance of identifying dynamic socio-ecological factors to enhance self-organization through analyzing collective human behaviors rather than imposing top-down rules. Accordingly, several recent works have reported how socio-ecological environments, societal network and reciprocity influence cooperation among individuals in a evolutionary perspective [26–28]. Individual cooperative behaviors in the eastern and western Germany have been studied in consideration of the different social histories of these regions [29, 30]. Authors find that subjects from the eastern region act more selfishly than those of the western region. Fishermen of individualistic lake-based fisheries are more competitive than those in collective sea-based fisheries, suggesting that daily practices with others in workplaces affect human behaviors and preferences [31].

The sustainability of natural resources is claimed to be endangered worldwide, as many countries are now moving toward more competitive environments. As socio-ecological environments are established to affect human nature, it is necessary to analyze how the ongoing modernization of competitive environments, i.e., “capitalism,” affects natural resource use. Despite their importance, no works have addressed these issues and thus this paper seeks to discuss how the degree of capitalism in societies characterizes individual prosociality, behaviors and CPR sustainability in the fields. To this end, we design and implement a set of dynamic CPR games and experiments in the two types of Nepalese areas, urban (capitalistic) and rural (non-capitalistic) areas. Nepalese areas are studied, because Nepal is characterized by relatively uniform ethnic, religious and cultural demographics, but has wide disparities between rural and urban areas with respect to daily life practices. The features of Nepal allow us to control for degrees of capitalism in our field experiments without experiencing confounding factors.

## Method and material

The field experiments of the CPR game incorporate resource dynamics in such a way that subjects with limited education understand. A group of 4 subjects is formed. Each subject is informed of the group size but not of the identities of the group members. Subjects are also told that the group members would remain the same. The resource stock at the beginning of each period is denoted by *x*_*t*_, where the subscript denotes time periods of *t* = 1, 2, …, and an initial stock size, *x*_1_, of 120 is given. At the beginning of each period *t*, subject *i* is asked to determine his/her individual harvest *y*_*i*,*t*_. The escapement, *s*_*t*_, is defined as $s_{t}=x_{t}-\sum_{j=1}^{4}y_{j,t}$ where $\sum_{j=1}^{4}y_{j,t}$ is the group harvest at period *t*. When *s*_*t*_ ≥ 0, then the individual payoff is *π*_*i*,*t*_ = *y*_*i*,*t*_. When *s*_*t*_ < 0, the individual payoff, *π*_*i*,*t*_, is $y_{i,t}=\frac{x_{t}}{4}$ for simplicity. The escapement, *s*_*t*_, is considered to be a remaining stock for each period *t* and determines the evolution of resource dynamics. The resource stock dynamics are specified as

$$x_{t+1}=\{\begin{array}{cc} 1.5s_{t}=1.5\left(x_{t}-\sum_{j=1}^{4}y_{j,t}\right)\; & s_{t}>0\\ 0 & s_{t}\leq 0. \end{array}$$ (1)

In this model, the next-period stock *x*_*t*+1_ grows up to a 50% increase in the escapement, and the game continues to the next period when *s*_*t*_ > 0 (the remaining stock is strictly positive). Otherwise, resource depletion results and the CPR game is terminated.

To simulate realistic conditions, we incorporate time discounting in the CPR games. We use total 20 chips in a box where 19 chips are white and 1 chip is red. The game can move to the next period when a representative of each group picks one chip and the chip is white. If a red chip is selected, the game is terminated for that group. This situation resembles the discount factor of *ρ* = 0.95 in terms of time preferences. In summary, our CPR games are terminated when a group depletes the resource, i.e., *s*_*t*_ ≤ 0, or when the red chip is selected by a group representative. With this setup, we are interested in identifying how many periods each group can sustain resource use in the games. The period at which each group terminates the game via resource depletion or chip selection is referred to as the “terminal period.” This is a measurement of the degree of sustainability.

This CPR game is designed to capture key factors of resource sustainability, reflecting some fundamental features of CPR utilization in the real world: (i) strategic uncertainty with anonymity, (ii) dynamic evolution of resources and (iii) time preferences of resource users. The game is framed within a resource utilization problem of multiple players on an infinite horizon, and it uses the following predictions of Nash equilibrium and Pareto optimality. One symmetric Markov perfect Nash equilibrium (potentially the simplest and played most frequently) states that each subject harvests the resource to exhaustion at an initial period. Pareto optimal allocation occurs when each subject in a group allows the resource to grow, and the group harvests the entire resource at once at the terminal period of budget and time constraints. The subjects are told that they may be asked to stop playing the game due to the “terminal period of budget and time constraints” if the game continues for too long.

The dynamic CPR field experiments were conducted in two types of Nepalese regions. The Kathmandu and Pokhara districts are urban, and the Chitwan and Parbat districts are rural (Fig 1). The Kathmandu and Pokhara districts are the first and second largest cities in Nepal, respectively, and these are the most highly populated areas in the country where most residents work in business, service and government sectors. The Chitwan and Parbat districts are rural areas consisting of small villages that are less densely populated where most residents work in the agriculture or forestry sectors. To ensure the random assignment of groups, subjects were selected from different cities and villages in cooperation with local NGOs and offices for each session. In using this approach, we avoided recruiting participants who knew one another.

**Fig 1:** The locations of fields: Kathmandu and Pokhara as urban areas and Parbat and Chitwan as rural areas.

A total of 528 subjects participated in this experiment, which is the maximum number of subjects that we could recruit under our time and budget constraints. As each group includes 4 subjects in the CPR game, the 67 groups and 65 groups of 268 and 260 subjects for the urban and rural areas were formed, respectively. In each session, 5 ∼ 8 groups convened in one place, and subjects were not allowed to communicate with one another. On average, each session of the CPR games and questionnaires lasted 3 hours. The subjects are told that the CPR game begins with an initial group token (initial resource stock) of 120 for each group, and that the next period would be reached as long as the resource is not depleted by the group members and as long as the red chip is not selected by the group representative. We described the resource and its dynamics using neutral terminology. The resource stock and escapement are expressed as “tokens” and “remaining tokens” for that given period, and the “next-period tokens” grow by 50% for the remaining tokens. We did not have access to computers or an internet connection in the field. The sessions were thus managed manually by experimenters and research assistants for each session.

At the start of each period, subjects were given the information on the group tokens and were asked to make an individual decision on how many tokens they would take. After the individual decisions were made, the participants were informed of the group harvest and of the remaining tokens. However, they were not informed of group members’ individual harvests. Unless no tokens were left, a representative of each group was randomly chosen to select one chip from a box with 19 white chips and 1 red chip. When a white chip was selected, the group moved to the next period. After completing the CPR games, we administered questionnaires on socio-demographic information and the social value orientation (SVO) game (adopting the “Slider Method”) for identifying subjects’ social preferences [32]. Subjects were paid real money based on the cumulative payoffs of their decisions made during the experiments including the SVO and CPR games in addition to a show-up fee in the local currency valued at US $2. Experimental rupees were converted to the Nepalese rupee (hereafter, NPR)at a rate of 1 experimental token = 2 NPRs. On average, NPR 500 was paid to the participants, which is nearly equivalent to $5.

### Ethics statement

This study was approved by the research ethics committee of Kochi University of Technology. Subjects provided their written consent to participate in this study.

## Results

We report a series of the questionnaire and experimental results with a focus on the rural and urban conditions with 65 and 67 groups of 260 and 268 subjects, respectively. Table 1 presents the summary statistics on the subjects’ socio-demographic information and on the experimental results. For the rural cohort, 38% of the participants are male with an average age of 34.5 years, while the urban cohort includes 58% men with an average age of 24.5 years. This result is attributed to the fact that many young men in the rural areas migrate to the urban areas or even to foreign countries for employment.

**Table 1:** Summary statistics.

Variables	Rural (65 groups, 260 subjects)					Urban (67 groups, 268 subjects)				
	Mean	SD^1^	Median	Min	Max	Mean	SD	Median	Min	Max
Age^2^	2.27	1.09	2.00	0.00	5.00	1.62	1.25	1.00	0.00	5.00
Gender^3^	0.38	0.49	0.00	0.00	1.00	0.58	0.49	1.00	0.00	1.00
Education^4^	9.58	3.40	10	1.00	16.00	13.07	3.57	16.00	1.00	16.00
Agriculture^5^	0.90	0.27	1.00	0.00	1.00	0.05	0.22	0.00	0.00	1.00
Income^6^	4.20	2.10	5.00	1.00	6.00	4.80	2.02	6.00	1.00	6.00
SVO^7^	0.76	0.43	1.00	0.00	1.00	0.39	0.49	0.00	0.00	1.00
Prosocial people in a group	3.03	0.93	3.00	1.00	4.00	1.57	1.08	1.00	1.00	4.00
Terminal periods	7.63	5.56	6.00	1.00	20.00	2.24	2.19	1.00	1.00	10.00
Individual harvest (payoff)^8^	143.14	443.54	47.50	12.00	3270.00	36.23	16.62	30.00	13.00	140.00
Prosocial individual harvest (payoff)^9^	174.49	505.67	53.00	12.00	3270.00	40.36	21.56	30.00	13.00	129.00

^1^ The “SD” stands for standard deviation.

^2^ Age is a categorical variable of {0, 1, 2, 3, 4, 5} where 0 is under 20, 1 between 20 and 30, 2 between 30 and 40, 3 between 40 and 50, 4 between 50 and 60. Finally, 5 is above 60 years old.

^3^ A dummy variable that takes 1 when the subject is male, otherwise 0.

^4^ Education represents years of schooling.

^5^ Agriculture is a dummy variable that takes 1 when a subject is stably employed or engage in agriculture/forestry sector as a main occupation. Otherwise 0.

^6^ It is a categorical variable of annual income measured by US dollar {1, 2, 3, 4, 5, 6}: 1. 0 ∼ 300, 2. 300 ∼ 600, 3. 600 ∼ 900, 4. 900 ∼ 1200, 5. 1200 ∼ 1500 and 6. more than 1500.

^7^ The “SVO” represents a dummy variable taking 1 (0) when a subject is prosocial (proself) based on SVO games.

^8^ Individual harvest (payoff) indicates the total harvest (payoff) a subject had from the dynamic CPR game.

^9^ Prosocial individual harvest (payoff) indicates the total harvest (payoff) a “prosocial” subject had from the dynamic CPR game.

With respect to education, more than 50% of the subjects in the urban areas have a university undergraduate degree (16 years of schooling as the median in Table 1), while the subjects in the rural areas possess 10 years of schooling as the median value. In regards to occupations, 90% and 6% of subjects in the rural and urban areas work in agriculture, respectively, implying that more than 90% of the urban subjects work in non-agricultural sectors such as the business, service and government sectors. Accordingly, household income is higher in the urban areas than in the rural areas. Overall, the summary statistics of socio-demographic information presented in Table 1 reflect the fact that urban areas are more capitalistic, providing non-agricultural employment and opportunities such as education. On the other hand, in the rural areas, individuals are less educated and tend to engage in agriculture and forestry.

Table 1 presents the subjects’ social value orientations (hereafter, SVOs) between the rural and urban areas where the SVO game was conducted to categorize subjects into a prosocial or proself group. First, a significant difference in SVOs is shown in the table, demonstrating that 76% of the subjects in the rural areas are prosocial, while only 39% of prosocial subjects are found in the urban areas. This difference affects the group composition of members based on SVOs between the rural and urban areas. In the rural areas, the average (median) number of prosocial members in a group is 3.03 (3), and it is 1.57 (1) for the urban areas. As one group includes 4 subjects, this is expected to affect how rural and urban groups harvest the resources. This SVO result shows that individuals are less prosocial in capitalistic areas, placing more emphasis on their own gains.

With respect to the terminal periods, the important results can be found for the measures of central locations and variability between the rural and urban areas. The median (average) terminal period is 6.00 (7.63) for the rural areas, while it is 1.00 (2.24) for the urban areas, implying that more than 50% of groups in the urban areas exhaust the resource or select a red chip at an initial period and never proceed to the 2nd period. On the other hand, most groups in the rural areas successfully continue the CPR game to more than 6 periods, and one group even reaches 20 periods of continuation. For the group achieving the “longest” play period, we asked the group members to stop the game due to time and budget constraints. The standard deviation for the rural areas (= 5.56) is much higher than that in the urban areas (= 2.19) (Table 1). These statistical findings are in line with the fact that the rural groups play the game for much longer than the urban groups.

Further, Table 1 shows the summary statistics of individual harvests (payoffs). The median (average) harvest is 47.50 (143.14) for the rural areas, while it is only 30 (36.23) for the urban areas. This is a clear evidence that urban subjects not only fail in sustaining the resources, but also end up having lower payoffs. Next, Table 1 also shows the summary statistics of “prosocial” individual harvests (payoffs) (Total harvests (payoffs) prosocial subjects had, and see Table 1 for the detailed definition). Interestingly, the median is 53 (174.49) for the rural areas, while it is only 30 (40.36) for the urban areas. This implies that prosocial subjects in the urban areas do not differ from general “urban” subjects with respect to harvests, but prosocial subjects in the rural areas perform better than general “rural” subjects.

Table 2 summarizes the frequency distributions of the terminal periods and of game termination via “red chip” selection. Red-chip terminations are more common for the rural areas than for the urban areas, with the overall percentage of red chips selected in the rural and urban areas amounting to 33% and 15%, respectively. This is consistent with the fact that the probability of red-chip termination increases with longer periods of play for the rural groups. In fact, only one red chip is selected among all 43 terminations at “terminal period 1” for the urban groups as shown in Table 2, implying that many urban groups (42 urban groups) terminate the game by exhausting the resources at the 1st period. On the other hand, the rural groups could have continued the game for much longer if there were no red-chip termination rule. Therefore, we believe that the significant gap in terminal periods between the rural and urban areas would exist irrespective of the red-chip termination rule.

**Table 2:** Terminal periods across the rural and urban areas.

Terminal periods	Frequency	Red chip	% of red chip
Urban areas			
1	43	1	2%
2	5	2	40%
3	6	2	50%
4	4	2	50%
5	3	2	67%
6	1	0	0%
7	2	0	0%
8	0	0	0%
9	2	0	0%
10	1	0	0%
Urban subtotal	67	10	15%
Rural areas			
1	7	0	0%
2	2	1	50%
3	10	3	30%
4	7	0	0%
5	4	3	75%
6	6	2	33%
7	3	1	33%
8	3	2	67%
9	3	3	100%
10	3	2	67%
11	0	0	0%
12	2	2	100%
13	2	2	100%
14	0	0	0%
15	1	0	0%
16	8	0	0%
17	1	1	100%
18	0	0	0%
19	2	0	0%
20	2	0	0%
Rural subtotal	65	22	33%

Fig 2 shows the corresponding frequency distributions where the vertical axis denotes the frequency and the horizontal axis denotes the terminal period. The distribution for the rural areas is broader than that for the urban areas, and the two frequency distributions are different from one another. In particular, the highest spike in the frequency distribution for the urban areas occurs in period 1, confirming that more than 50% of urban groups terminate the game at an initial period. For the post-questionnaires, we include the following question: “how did you want to play?” A considerable number of urban subjects answered to this question as follows: “I really wanted to play the game for longer, but I was not sure whether the other group members were motivated to do the same.” This type of answer was given by 51% of the urban subjects. It appears that many urban subjects recognize some potential benefits of playing the game for longer. However, they did not actually restrain their harvests for continuation even at an initial period due to their concerns about other members. To confirm the difference in frequency distributions between the rural and urban areas, we conducted a Mann-Whitney test. The result shows that the frequency distributions differ from one another at a 1% level of statistical significance.

**Fig 2:** Frequency distributions of terminal periods between rural and urban areas. The frequencies of terminal periods between the urban (the left) and rural (the right) areas are shown separately.

We characterize resource sustainability in the dynamic CPR games by running regression of the terminal periods where the rural dummy, SVO and socio-demographic information are taken as independent variables. As the terminal periods take positive integers, a Poisson regression is employed in our analysis. The Poisson regression model can be specified as:

$$Y_{j}=\beta_{0}+\beta_{1}X_{j}+\beta_{2}R_{j}+\beta_{3}Z_{j}+\epsilon_{j},$$ (2)

where *j* is a group index from 1, …, *n*, *Y*_*j*_ is the explanatory variable (terminal periods) for group *j*, *X*_*j*_ is a number of prosocial members in group *j*, *R*_*j*_ is a regional dummy variable taking 1 if the region of group *j* is rural, otherwise 0, and **Z**_*j*_ is a vector of other socio-demographic independent variables that may be assumed to characterize the terminal periods *Y*_*j*_. Finally, *ϵ*_*j*_ is an error term. The parameter *β*_*i*_ for *i* = 0, 1, 2 is a set of coefficients for an intercept, *X*_*j*_ and *R*_*j*_, respectively. The *β*_3_ is a vector of coefficients for other independent variables **Z**_*j*_. We are interested in estimating the coefficients of *β*_1_ and *β*_2_, but we cannot interpret them as they are given. The marginal effect of the number of prosocial members in a group can be approximated by 100 ⋅ *β*_1_ which is interpreted as the percentage change. The marginal effect of the regional dummy (percentage change) is derived from a formula of exp(*β*_2_) − 1 (See, e.g., Wooldridge [33]).

Table 3 reports the estimated coefficients and their respective standard errors with statistical significance. Model 1 includes the number of prosocial members in a group and the regional dummy as independent variables. The results reveal that both independent variables exhibit a statistical significance of 1% and positively affect the terminal periods. More specifically, the expected terminal period increases by 68% with an increase of prosocial members in a group, holding other factors fixed. The expected terminal period for the rural areas is interpreted to be approximately 45% higher than that for the urban areas, holding other factors fixed. As mentioned earlier, the marginal effect of the regional dummy variable can be approximated by the following formula: exp(.37) − 1 ≈ 0.448 ≈ 45%. These marginal effects are considered to be economically significant, illustrating the strong effects of member prosociality and of the regional dummy. As the regional dummy used in our analysis is considered to represent the degree of capitalism, we conclude that resource sustainability tends to be compromised as societies become more capitalistic.

**Table 3:** Poisson regression for the terminal periods in the dynamic CPR games.

	Model 1	Model 2
# of prosocial members in a group	0.68*** (0.041)^1^	0.65*** (0.044)
Regional dummy	0.37***	0.49*** (0.108)
Av. income in a group		−0.29 (0.042)
# of males in a group		0.077** (0.039)
Av. education in a group		−0.0045 (0.021)
Av. age in a group		−0.077 (0.070)
Constant	−0.55*** (0.13)	−0.37 (0.44)
Wald χ^2^	333.08***	530.86***
Pseudo *R*^2^	0.46	0.46

^1^ Numbers in parentheses are robust standard errors

***significant at the 1 percent level,

**significant at the 5 percent level and

*significant at the 10 percent level.

For the robustness check, we run another Poisson regression by including other independent variables of individual characteristics as shown in model 2 of Table 3, the average income, the number of males, the average education level and the average age for each group in both areas. The main results of model 2 do not differ from those of model 1. Rather, the economic significance of the estimated coefficient for the regional dummy increases, while it almost remains the same for the number of prosocial members in a group. The estimated coefficients for the number of prosocial members in a group and the regional dummy are still statistically and economically significant. The expected terminal period is interpreted to increase by 65% with an increase in prosocial members in a group. Likewise, the expected terminal period for the rural areas is estimated to be roughly 63% higher than that for the urban areas (The marginal effect of a regional dummy = exp(0.49) − 1 ≈ 0.63).

It is also observed that average income, average education and average age have no significant effects. An exception is that the number of males in a group that shows a positive effect with statistical significance of 5%. However, the magnitude is 7.70%, which could be considered small in comparison to the regional effect and social preferences. This result may derive from gender inequality in the society as Nepal is a highly male-dominated society. Past literature has also revealed that women are less cooperative with outgroup members than men [34]. We attempted to create alternative specifications for the Poisson regression. However, the results with respect to the number of prosocial members in a group and the regional dummy do not change significantly. We confirm that these two variables remain statistically and economically significant, irrespective of the specifications used in the models. The SVO and the degree of capitalism (regional dummy) are key determinants of resource sustainability.

The SVO is a good proxy for individual social preferences, and our SVO results are intuitive in the sense that more prosocial subjects in a group lead to better resource sustainability outcomes. On the other hand, our results for the regional dummy raise the following question. What does the regional dummy truly capture in the regression? In this paper, we define capitalism as the ongoing modernization of competitive societies. Urban areas examined in the field experiment (e.g., Kathmandu) are considered to be capitalistic societies, rapidly developing in a competitive fashion. By contrast, rural areas such as the Chitwan district are still home to agrarian and traditional societies.

Urban areas such as Kathmandu have attracted a large number of migrants from other areas of Nepal. Individuals migrate to urban areas because they imagine that better opportunities for safety, education and employment are provided in these areas. In reality, however, urban areas in Nepal have become denser, and individuals are required to compete with others for survival in business, service and government sectors by utilizing their skills and education. In many cases, individuals do not know who their neighbors are with their busy lives. Simply put, life in current Nepalese urban areas does not require individuals to interact or to cooperate with neighbors and others on a daily basis. Recall that more than half of urban subjects answered in our questionnaire surveys “I really wanted to play the game for longer, but I was not sure whether the other group members were motivated to do the same.” This trend represents the general assumptions urban subjects possess about how other people behave.

In the rural areas, most individuals still engage in agriculture and in natural resource management based on indigenous knowledge and traditional practices where cooperation and sharing are quite common among individuals. For instance, *Mela pat* and *Parma* are well known as voluntary and cooperative farming practices that prevail in rural Nepalese culture. Individuals exchange or offer farming and forestry services without monetary rewards. Such forms of voluntary cooperation remain common of Nepalese rural areas, as rural residents are vulnerable to natural uncertainties and calamities, and cannot sustain their lives without mutual cooperation. We suspect that such regular human network linkage through daily interaction in Nepal shape rural individuals’ preferences, customs, norms, assumptions about others through for sustainably managing resources.

In our dynamic CPR games, each subject in a group does not know the identity of other group members, and cannot infer how other members behave. That is, each subject needs to decide what to do under the poor information environment. In such a case, it is claimed that people follow what they have experienced, learned and observed from others in their daily life, and their behaviors shall be dominated by not only individual preferences (SVOs) but also conformity for proper actions that people have developed [11, 35]. In particular, it is our belief that the individual decisions and outcomes in the 1st period of the dynamic CPR games shall be influenced by such conformity. From the 2nd period onward, each subject confirms and/or adapts her actions to updated conformity, following the observations in the previous periods. The conformity people possess based on their daily life appears to be very different between urban and rural areas, reflecting a huge discrepancy of 1st-period outcomes and the strong effect captured by the regional dummy in the regression analyses.

In summary, the differences in daily practices of cooperation and competition for survival or for earning incomes between the rural and urban areas appear to affect individuals’ preferences, customs, social norms on resource use, assumptions about others, etc in collective CPR settings. The regional dummy is considered to capture important factors other than the SVO. Following the previous arguments that social environments affect individual preferences and behaviors [31, 36–41], our field experiment serves as a first attempt to demonstrate that both the SVO and other factors captured by the degree of capitalism (regional dummy) are important for resource sustainability. This analysis shows that resource sustainability will be compromised by changes in human nature through interactions between individuals, as societies develop in capitalistic ways. This implies that individuals may be losing their coordination abilities to solve social dilemmas of resource sustainability in capitalistic societies.

## Conclusion

This experiment has analyzed resource sustainability in a dynamic setting with respect to the degree of capitalism and social preferences. We find that the proportion of prosocial individuals in the urban areas is lower than that in the rural areas, and urban residents deplete resources more quickly than rural residents. The composition of proself and prosocial individuals in a group and the degree of capitalism (rural vs. urban) are identified as two central factors, such that an increase in prosocial members in a group or the regional change from the urban to the rural improve resource sustainability by approximately 65% and by 63%, respectively. Overall, this paper shows that when societies evolve into more capitalistic environments, the sustainability of common pool resources tends to be lost via changes in individual preferences, social norms, customs and assumptions about others through the ways of human interactions. That is, individuals may be losing their coordination abilities in managing social dilemmas of resource sustainability in capitalistic societies.

We note some limitations of our study. This research does not fully address the details of rural-specific effects on the sustainability of common pool resources. In reality, rural-specific effects might not only compose of the ways of human interactions or human network but in a daily life there could be other factors, such that it hold strong social capital or conformity among them. In the future, we should collect more detailed data about human interactions and other possible factors that may represent the differences between rural and urban areas. If such rich data are successfully collected, new methodologies such as social network methods can be utilized to analyze network effects in resource utilization. It is also very important to ensure external validity of our findings by conducting further experiments in the future. Shahrier et al. [42] show that a larger proportion of prosocial people are found in rural areas than urban areas in Bangladesh, which is consistent with our result. We expect that the same type of qualitative results with our CPR experiments shall be confirmed in different countries and contexts. These caveats notwithstanding, it is our belief that this field experiment is an important first step to characterize resource sustainability in relation to the degree of capitalism and social preference. Our results clearly suggest that new institutions or devices are necessary for urban people to manage CPRs in a sustainable way.

## Supporting information

S1 File Excel “CPRs” data file. It contains all the necessary data to replicate the statistical and regression results presented in this paper.
(XLSX)
